RETRACTED

# Novel Therapeutic Mechanism of Adipose-Derived Mesenchymal Stem Cells in Osteoarthritis via Upregulation of BTG2

**DOI:** 10.1155/2022/9252319

**Published:** 2022-10-15

**Authors:** Qinyan Yang, Li Jin, Qian Ding, Wei Hu, HaiBo Zou, Mingming Xiao, Keyuan Chen, Yue Yu, Jin Shang, Xiaolun Huang, Yizhun Zhu

**Affiliations:** ^1^State Key Laboratory of Quality Research in Chinese Medicine & School of Pharmacy, Macau University of Science and Technology, Taipa, China; ^2^Department of Hepatabiliary and Pancreatic Surgery Center, Cell Transplantation Center, Sichuan Provincial People's Hospital, University of Electronic Science and Technology of China, Chengdu, China; ^3^Chinese Academy of Sciences Sichuan Translational Medicine Research Hospital, Chengdu 610072, China; ^4^Clinical Immunology Translational Medicine Key Laboratory of Sichuan Province, Sichuan Provincial People's Hospital, University of Electronic Science and Technology of China, China

## Abstract

**Background:**

Osteoarthritis (OA) is a debilitating and degenerative joint disease, which is characterized by progressive destruction of articular cartilage. Mesenchymal stem cells (MSCs) have been implicated in the treatment of OA. However, the function of adipose-derived MSCs (AD-MSCs) in OA and its underlying mechanism remain obscure.

**Aim:**

We aimed to explore the function of AD-MSCs in OA and investigate its potential regulatory mechanism.

**Methods:**

A guinea pig model of OA was constructed. AD-MSCs injected into the articular cavity of OA guinea pigs were viewed by *in vivo* bioluminescence imaging. The effect of AD-MSCs on the gonarthritis of OA guinea pigs was evaluated through both macroscopic and microscopic detections. The detailed molecular mechanism was predicted by GEO databases and bioinformatics tools and then verified via mechanism experiments, including ChIP assay, DNA pulldown assay, and luciferase reporter assay.

**Results:**

AD-MSCs had a significant positive therapeutic effect on the gonarthritis of the OA model, and the overall effects of it was better than that of sodium hyaluronate (SH). B-cell translocation gene 2 (BTG2) was significantly downregulated in the articular cartilage of the OA guinea pigs. Furthermore, BTG2 was positively regulated by Krüppel-like factor 4 (KLF4) in AD-MSCs at the transcriptional level. AD-MSCs performed an effect on KLF4 expression at the transcriptional levels.

**Conclusion:**

AD-MSCs suppresses OA progression through KLF4-induced transcriptional activation of BTG2. Our findings revealed an AD-MSCs-dominated therapeutic method for OA.

## 1. Introduction

Osteoarthritis (OA) is the most prevalent musculoskeletal disease and a significant healthcare burden on the public since it attacks about 10% of men and 18% of women more than 60 years old [1]. Articular cartilage degradation, subchondral bone sclerosis, inflammation, and osteophyte formation are key characteristics of OA [2]. Oxidative stress, a major cause of chronic inflammation, is increased in OA cartilage. It occurs based on an imbalance between the production of reactive oxygen species (ROS) and their removal by the antioxidant defense system [3]. Due to inadequate blood supply of articular cartilage and high differentiation of chondrocytes [4], the therapeutic efficacy of OA is always limited.

RETRACTED

Mesenchymal stem cells (MSCs) are multipotent adult cells that can be isolated from various adult or neonatal tissues, which has been used in the clinical management of OA [5]. For example, the intra-articular injection of bone marrow-derived MSCs (BM-MSCs) contributes to the regeneration in knee osteoarthritis [6]; Human synovial fluid-derived MSCs (SF-MSCs) have the potential to affect cartilage repair in OA [7]. Nowadays, the mechanisms of BM-MSCs and SF-MSCs in OA have been widely reported [8–11]. In addition to BM-MSCs and SF-MSCs, many studies have also discussed the function of adipose-derived MSCs (AD-MSCs) in OA [12, 13]. As reported previously, small molecules like miRNAs in extracellular vesicles from AD-MSCs may be associated with OA pathogenesis [14]. Besides, AD-MSCs could regulate the expression of inflammatory cytokines and bone morphogenetic proteins to ameliorate OA [15]. However, the detailed mechanism of AD-MSCs in attenuating OA progression remains unknown.

To probe into the potential mechanism by which AD-MSCs regulated OA, we established a guinea pig model of OA. From the GEO database, we analyzed OA-related genes and selected BTG2 as the further research object. Subsequently, we conducted mechanism investigation to verify the involvement of KLF4-induced BTG2 in AD-MDCs-mediated OA. RNA-induced oxidative stress is closely related with disease progression [16, 17]. In this study, we also detected the effect of BTG2 on oxidative stress. In a word, our current study unveiled a novel potential molecular mechanism of AD-MSCs functioning in the treatment of OA.

## 2. Materials and Methods

### 2.1. Animal Model of OA

Fifty-six guinea pigs weighing 350-400 g were randomly divided into four groups after one week of adaptive feeding. The eight guinea pigs from the first group were sham-operated (control group without any other treatment subsequently), and the other three groups of 48 guinea pigs were received medial meniscus transection (MMT): the skin was cut on the medial side of the knee joint, the medial ligament was cut for exposing the medial meniscus, and then the meniscus was cut from the incision and sutured. After two weeks of regular feeding, three groups of guinea pigs that underwent MMT were renamed according to indicated treatments: MSC group (experimental group), sodium hyaluronate (SH) group (Bausch & Lomb, China; positive control group), and normal saline (NS) group (Double Crane, China; negative control group). For the MSC group, 100 *μ*L CFDA-labeled AD-MSC suspension (1 × 10^7^ cells/mL) of P5 generation was injected into the joint cavity; for the SH group, 100 *μ*L SH (0.5 mL/5 mg) was injected into the joint cavity; for NS group, 100 *μ*L NS was injected into the joint cavity. There were 8 guinea pigs in the control group and 16 in each of the rest three groups. Then, half of the animals from each group were sacrificed three weeks after indicated injections, and the other half were sacrificed after eight weeks of injection. Afterwards, the joints were collected, and the articular cartilages were observed and photographed. Three individuals scored the cartilage defects independently to evaluate the articular cartilage damage, with the joint score scale shown in Table 1. And then, the cartilages were subjected to HE staining, safranin O-fast green staining, toluidine blue staining, Sirius red staining, and immunocytochemistry for type II collagen (Col2) as described [18, 19]. All procedures were carried out in accordance with the guidelines by the Division of Animal Control and Inspection of the Department of Food and Animal Inspection and Control of Macau and were approved by the Animal Care and Use Committee (ACUC) of the Macau University of Science and Technology (SCXK-2018-0010).

RETRACTED

### 2.2. Magnetic Resonance Imaging (MRI) of Knee Joints of OA Guinea Pigs

At the 3^rd^ and 8^th^ week after the construction of the guinea pig model of OA, BioSpec70/20USR MRI (Bruker, Germany) was performed on a 7.0 T MRI system using a 40-mm mouse body coil. Parameters for the T2 imaging sequence were set as TR = 2100 ms, TE = 40 ms, FOV = 20 mm × 20 mm, layer stick = 0.5 mm, and MTX = 200 × 200. T2 relaxation time was calculated from the sagittal plane through the center of the cartilage repair site using the Bruker Para Vision 6.0 system. MRI images showed the filling of cartilage injury, and the T2_mapping sequence was used to measure the regeneration of cartilage defect at the 3^rd^ and the 8^th^ week after injection. Guinea pig joint samples were imaged for the control, NS, and SH groups, and samples were observed for the MSC group.

### 2.3. Bipedal Balance Pain Testing

To analyze the weight distribution of both feet, guinea pigs were put in an angled plexiglass chamber and assessed via a bipedal balance tester (Stoelting Co; Wood Dale, IL, USA). In detail, each hind paw of guinea pigs was put on a separate force plate, with force exerted by each hind limb (in grams) determined within 5 seconds. Each guinea pig was subjected to three independent tests, and the data were calculated as the average value. The sensitivity of the injured side is uniformly expressed as the injured/non-injured weight percentage. The tests were carried out 3 or 8 weeks after indicated injections before the animals were sacrificed.

RETRACTED

### 2.4. Cell Culture

AD-MSCs were isolated and extracted by collagenase method. Wash the adipose tissue, and add 0.75 mg/mL type I collagenase solution for 30 minutes at 37°C. Gently discard the supernatant without disturbing the precipitated cells, resuspended with an appropriate amount of normal saline and mixed well. Centrifuge at room temperature 300 g for 10 minutes. Carefully suck off the supernatant. Suction pipette head should be placed on the upper liquid level of the centrifuge tube to thoroughly remove grease. Add normal saline to the precipitate and resuspended the mixed cells. Filter the cell suspension with a 100-*μ*m cell filter, followed by the criteria [20], in Mesenchymal Stem Cell Basal Medium (MSCBM) (Dakewe, Chengdu, China) with 5% Knockout Serum Replacement (KSDR) (EliteGro, TX, USA). Primary cells were defined as passage 0, and cells passaged to the fifth generation were used for *in vitro* experiments (Chengdu Baimeisen Biological Technology Co. Ltd. provided the AD-MSCs and culture methods). The identification of AD-MSCs was described in Figure S1. The human embryonic kidney cell (HEK293T) cell line obtained from American Type Culture Collection (ATCC, Manassas, VA, USA) was cultivated in RPMI-164 medium with 10% FBS. The above cells were grown in a humid incubator which was set with 5% CO_2_ and 37°C.

### 2.5. Quantitative Real-Time Polymerase Chain Reaction (qRT-PCR)

The qRT-PCR analysis was performed as previously described [21]. Total RNA was extracted from tissues and cells with TRIzol reagent. A PrimeScript-RT Kit was applied to reverse transcribe the total RNA to synthesize cDNA. qRT-PCR was performed with SYBR Green PCR Kit. RNA expression was calculated by 2^-*ΔΔ*Ct^ method and normalized to GAPDH.

### 2.6. Measurement of ROS Production and Superoxide Dismutase (SOD) Production

Cellular ROS Assay Kit (ab113851, Abcam, Cambridge, MA, USA) was utilized to detect intracellular ROS levels as per the manufacturer's instructions. SOD activity was measured using SOD Determination Kit (19160, Sigma-Aldrich, St. Louis, MO, USA) according to the manufacturer's instructions [16]. The level of SOD (U/mg protein) was examined using Synergy-2 microplate reader (BioTek, Winooski, VT, USA).

RETRACTED

### 2.7. Flow Cytometry Analysis

Flow cytometry was conducted as previously described [22]. AD-MSCs at the fifth passage reached 80% confluence and were trypsinized, washed, centrifuged, and resuspended in PBS. Subsequently, AD-MSCs were incubated with antibodies against CD90, CD105, and CD73 and the negative control Neg CKTL, which were then subjected to flow cytometry analysis.

### 2.8. Chromatin Immunoprecipitation (ChIP) Assay

ChIP assay was performed to validate the interaction between KLF4 and BTG2 promoter by using the ChIP assay kit as previously described [23]. AD-MSCs were first cross-linked in 4% paraformaldehyde and then sonicated into chromatin fragments of 200-1000 bp, which were incubated with anti-KLF4 or negative control anti-IgG. Subsequently, the chromatin was incubated with magnetic beads. Finally, the precipitated DNAs were purified and analyzed by qRT-PCR.

### 2.9. Western Blot Assay

Total proteins were tissues or cells using RIPA lysis buffer (Beyotime Institute of Biotechnology, China). Protein concentration was determined by using BCA Protein Assay Kit (Abcam, China) according to the manufacturer's instructions. After separation by PAGE, total proteins were transferred onto PVDF (Millipore, USA) membranes and blocked by 5% BSA for 1 h at room temperature. Then, PVDF membranes were incubated with primary antibodies at 4°C overnight. The primary antibodies were as follows: BTG2 (1 : 1000), KLF4 (1 : 1000), and actin (1 : 2000) (Abcam, USA). Next, the membranes were washed with TBST three times and incubated with secondary antibody HRP-labeled goat antirabbit IgG for 1 h at room temperature. Protein expressions were determined using Uvitec Alliance software (Eppendorf, Germany).

### 2.10. Luciferase Reporter Assay

To verify the bond of KLF4 to BTG2 promoter, the BTG2 promoter contained KLF4 binding sites, or mutant binding sites was separately subcloned into pGL3 luciferase reporter vector to build the constructs. The constructs were cotransfected with si-KLF4 or si-KLF4 into HEK293T cells. The luciferase activities were analyzed utilizing the Dual-Luciferase Reporter Assay System [24] and normalized to Renilla luciferase activity.

### 2.11. DNA Pulldown Assay

As previously described [25], DNA pulldown assay was conducted to prove the affinity of KLF4 to BTG2 promoter. Cell lysates and BTG2 promoter-specific biotinylated probes were incubated for 2 h at room temperature with streptavidin–agarose beads to form DNA-protein-beads complexes. The complexes were then separated on a magnetic rack. The pulled-down complex was washed six times with 1 mL ice-cold tris-buffered saline and eluted in 80 *μ*L protein elution buffer at 95°C for 5 min. Proteins were separated by gel electrophoresis and measured by western blot.

RETRACTED

### 2.12. Statistical Analysis

For animal experiments, *N* = 4 in the control group and *N* = 8 in other three groups. For cell experiments, *N* = 3 in each group. Each independent experiment was operated at least three times to ensure the accuracy of the results, and experimental data of three or more replicates were illustrated as the means ± SD. The statistical analysis was made by using SPSS 19.0 software with the method of Student's *t*-test or one-way ANOVA. The data were regarded as statistically significant when *P* < 0.05.

## 3. Results

### 3.1. AD-MSCs Exhibit Therapeutic Effect on Guinea Pig Model of OA

To investigate the impact of AD-MSCs on OA, we established an OA model in guinea pigs. As shown in Figure 1(a), AD-MSCs marked with CFDA were observed in the joint area, and cells were concentrated on the articular cartilage surface. After injections, all of the guinea pigs were observed for 3 weeks. It was found that the action competence of guinea pigs treated with MMT gradually weakened. Next, we discovered from the bipedal balance pain testing data that the pain sensitivity of guinea pigs was evidently strengthened in NS groups than other groups after 3 weeks, and such eigenvalue was then partly recovered after 8 weeks. The MSC group looked a little better than the SH group after 3 weeks (although not significant). However, the results seemed to be similar after 8 weeks between the guinea pigs injected with AD-MSCs and those injected with SH (Table 1) (Figure 1(b)).

Additionally, MMT-induced articular cartilage damage in OA guinea pigs was relieved by treatment with AD-MSCs or SH after 3 weeks and even after 8 weeks. Compared with the control group, the knee cartilage of guinea pigs in the NS group was damaged after 3 weeks, with an uneven surface and terrible inflammatory exudation beneath. Additionally, the SH group and the AD-MSCs group had partial cartilage defects. The cartilage surface was more intact in the AD-MSCs group than in the SH group after 3 weeks. After 8 weeks, the knee cartilage in the NS group was severely damaged, even with bone corrosion. In comparison, the cartilage in the SH group appeared to be partially defective and imperfection. The AD-MSCs group showed remarkable changes. With most of the articular cartilage covered and only left a tiny loss of ostiole, the damage seemed to be repaired after 8 weeks (Figure 1(c)).

To compare the joint damage in different groups, the OA gross joint score system was used to evaluate the injured joint. It turned out that the joint damage in AD-MSCs group was remarkably repaired. Both the AD-MSCs group and the SH group exhibited higher OA scores compared with the NS group after 3 weeks. After 8 weeks, OA score in the AD-MSCs group and the SH group was also higher than the NS group (Figure 1(c)). In sum, AD-MSCs exhibit therapeutic effect on guinea pig model of OA.

RETRACTED

### 3.2. AD-MSCs Repair the Cartilage of the Guinea Pig OA Model

The above results indicated that the therapeutic effect of AD-MSCs on OA was better than SH treatment. However, the specific difference between AD-MSCs and SH treatments was unclear, especially the results after 8 weeks. According to the MRI images, we observed that the cartilages of knee joints were indeed injured after MMT treatment at both 3 and 8 weeks, and AD-MSCs or SH injection could lead to the regeneration of cartilage defects.

Normal articular cartilage surface is clear and smooth. Its morphology on MRI is intact, and its thickness is uniform. MRI image of the AD-MSCs group showed that its articular cartilage was similar to that of the control group after 3 weeks. The cartilage of the SH group was a little thin, while the integrity was fair. Nonetheless, there was still some inflammation in the joint cavity of SH group. Furthermore, MRI image of NS group showed a largest cartilage wear, a serious joint cavity deformation with osteolysis, and a severe inflammatory reaction after 3 weeks (Figure 2(a)).

The results in the SH group after weeks were similar to those after 3 weeks, with thinner cartilage, fair integrity, and some inflammation in the joint cavity. The cartilage of the AD-MSCs group was similar to the SH group, and the cartilage was repaired and intact. The NS group had apparent cartilage damage and severe joint cavity deformation. The articular surface was severely worn, and the medial tibial plateau and femoral joints were incomplete. Even the subchondral bone was lost with osteolysis (Figure 2(b)). Altogether, AD-MSCs treatment for OA is more effective than SH treatment.

### 3.3. AD-MSCs Have Therapeutic Effects on the Gonarthritis Cartilage Tissues in OA Guinea Pig

We further evaluated the microscopic changes induced by AD-MSCs on the gonarthritis in OA guinea pigs through the macroscopic observation. As shown in HE staining, the articular cartilage tissues were evidently damaged in guinea pigs treated with MMT followed by NS treatment, while SH and AD-MSCs treatments repaired MMT-induced damages after 3 weeks and 8 weeks. Articular cartilage defects were similar in the SH and AD-MSCs groups, and both groups were superior to the NS groups. Furthermore, the loss of cartilage matrix in the NS group was severe, accompanied by the infiltration of some inflammatory cells after 3 weeks (Figure 3(a)). Compared with the control group, there were articular cartilage defects in all other three groups after 8 weeks. The articular cartilage defects in the SH group and the AD-MSCs group were partially repaired with little loose structure and morphological changes. Although the inflammatory state subsided after 8 weeks, there was no significant repair of articular cartilage defect in the NS group (Figure 3(a)).

RETRACTED

Similar results were also observed through safranin O-fast green staining. After 3 weeks, the staining of the SH group was deeper than that of the AD-MSCs group, despite the results in the AD-MSCs group being significantly better than the NS group. The NS group had little staining because of the partial loss of cartilage (Figure 3(b)). However, the cartilage defects in the AD-MSCs group were repaired better than that in the SH group after 8 weeks. In the NS group, cartilage damage and loss were obvious, and no repair traces were found (Figure 3(b)).

Furthermore, toluidine blue staining was performed to detect the content of glycosaminoglycan (GAG), an important component of the cartilage extracellular matrix (ECM). Staining of the articular cartilage of the knee joint in the AD-MSCs group was stratified. The staining of the SH group was inferior to that of the AD-MSCs group. Besides, the NS group took less color after 3 weeks, even no blue-colored part was observed after 8 weeks (Figure 3(c)).

Sirius red staining was further used to visualize significant collagen matrix deposition in the regenerated tissues of each group. Under the polarized light microscope, there was mainly yellowish green in the control group after 3 weeks and 8 weeks. However, the AD-MSCs group appeared richly bright in red, yellow, and green due to active tissue repair, especially lasted after 8 weeks. The SH group showed yellow and green, with loose tissue arrangement and partial reticular structure after 3 weeks and 8 weeks. Tissue repair degree weakened obviously after 8 weeks. The NS group showed dully green color and weak refraction after 3 weeks and 8 weeks. In terms of the degree of the collagen matrix deposition of gonarthritis in guinea pigs after 3 weeks and 8 weeks, the tendency of four groups was MSC>SH>NS>control (Figure 3(d)).

Immunocytochemistry staining of Col2, which was explicitly expressed in newborn tissues and articular cartilage tissues, was performed in four groups. Col2 was widely localized in the intercellular space and extracellular matrix in the SH group, especially in the AD-MSCs group after 3 weeks and 8 weeks. In contrast, the staining of the NS group was slight, and the cartilage tissue of NS group damaged severely after 3 weeks and 8 weeks compared with the control group (Figures 3(e)). These data indicated that AD-MSCs have better therapeutic effects on the gonarthritis cartilage tissues of OA guinea pigs than SH treatment.

RETRACTED

### 3.4. The Effects of AD-MSCs on the Changes of Inflammatory-Associated Cytokines

The infiltration of inflammatory cells was observed in the pathological section and staining. To identify the inflammation conditions, we tested the levels of inflammation-associated cytokines in four groups. As a result, we found that the contents of proinflammatory cytokines including IL-1*β*, TNF-*α*, IL-1, IFN-*γ*, and IL-13 in the serum and synovial fluid were enhanced in the NS group, whereas such enhancement was offset by AD-MSCs or SH treatment for both 3 and 8 weeks (Figures 4(a)–4(e) and Figure S2A-S2E). Meanwhile, the decreased levels of anti-inflammatory factors (TGF-*β* and IL-4) induced by NS treatment was enhanced by AD-MSCs or SH treatment for both 3 and 8 weeks (Figures 4(f) and 4(g) and Figure S2F-S2G). Likewise, the levels of MMP-1 and MMP-13 were changed along with proinflammatory cytokines in the serum and synovial fluid (Figures 4(h) and 4(i) and Figure S2H-S2I). As two OA-related factors, ADAMTS4 and ADAMTS5 were enhanced in the NS group compared to the control group and were reduced by AD-MSCs and SH injection for either 3 or 8 weeks (Figures 4(j) and 4(k) and Figure S2J-S2K). Similarly, the articular cartilage repair factor IGF-1 was also highly expressed in the NS group, but this tendency was partly counteracted in the AD-MSCs group and the SH group (Figure 4(l) and Figure S2L). All the data showed that AD-MSCs alleviates the gonarthritis in OA guinea pigs.

### 3.5. BTG2 Is Significantly Downregulated in the Articular Cartilage of OA Guinea Pig

Subsequently, we explored the detailed regulatory mechanism of AD-MSCs in treating OA. Searching from the GEO database (https://www.ncbi.nlm.nih.gov/geo/), we selected 9 differential expressed genes (logFC< -1.0) related to OA progression from the datasets GES12021, GSE55235, and GES55457, including MCL1, GRB10, VEGFA, BTG2, APOLD1, SIK1, GADD45B, KLF9, and TNFAIP3 (Figure 5(a)). Trough qRT-PCR analysis, we found that BTG2 exhibited the most significant declined expression in the OA group in comparison with the Sham group (Figure 5(b)). Therefore, we chose BTG2 for further studies. At the same time, BTG2 expression was markedly increased in the AD-MSCs group and the SH group, especially in the AD-MSCs group (Figures 5(c) and 5(d)). Since oxidative stress is closely related with OA progression, we also detected the oxidative stress in the chondrocytes of the OA model with BTG2 overexpression. It was uncovered that ROS accumulation was decreased after overexpression of BTG2 (Figure S3A). Meanwhile, the SOD activity was enhanced in BTG2-overexpressed group (Figure S3B). In sum, BTG2 is downregulated in the articular cartilage of OA and may suppress oxidative stress.

RETRACTED

### 3.6. KLF4 Transcriptionally Induces BTG2 in Chondrocytes

Furthermore, we explored the upstream molecular mechanism of BTG2 in chondrocytes of the OA model. Transcription factors (TFs) are crucial regulators of their target genes. Hence, we firstly applied hTF target (http://bioinfo.life.hust.edu.cn/hTFtarget#!/) to predict BTG2-associated TFs and then intersected this subset with GES12021, GSE55235, and GES55457 (*P* < 0.05, logFC <0) to select potential TFs functioned in OA. As a result, 10 candidates, including JUN, ATF3, BHLHE40, EGR1, MYH11, MYC, JUNB, KLF9, KLF4, and BRD4, were screened out (Figure 6(a)). Among these candidates, BHLHE40, MYH11, and KLF9 have not been reported in OA yet, and KLF4 has been recognized as a suppressor of OA [26, 27]. Next, we overexpressed these four candidate TFs and found that KLF4 exhibited the most significant effect on BTG2 expression (Figure 6(b)). In addition, BTG2 expression was notably decreased after KLF4 interference (Figure 6(c)). Next, ChIP data manifested the strong enrichment of BTG2 promoter in the anti-KLF4 group compared with the control anti-IgG group (Figure 6(d)). The binding sites between KLF4 and BTG2 promoters predicted using the JASPAR tool (http://jaspar.genereg.net/) are exhibited in Figure 6(e). Luciferase reporter assay indicated that after KLF4 downregulation, the luciferase activity of pGL3 vector with full-length BTG2 promoter, 1898-1909-mutated BTG2 promoter, or 1831-1842-mutated BTG2 promoter was declined, while that of pGL3 vector containing BTG2 promoter with mutated 54-65 fragment was almost unchanged (Figure 6(f)). It was also verified by DNA pulldown assay that KLF4 could be pulled down by the probe biotinylated with full-length BTG2 promoter rather than that with the BTG2 promoter contained mutated 54-65 fragments (Figure 6(g)). Furthermore, the protein level of KLF4 among the different animal groups has been examined by western blotting. The results showed that KLF4 expression was markedly increased in the AD-MSCs group and SH group after 3 weeks and 8 weeks, especially in the AD-MSCs group after 8 weeks (Figure 6(h)). The above findings indicated that KLF4 is a transcriptional activator of BTG2.

## 4. Discussion

OA represents the most prevalent chronic joint disease characterized by the degradation of articular cartilage and remodeling of the underlying bone [28]. MSCs have been reported as an important treatment option for OA [29]. Besides, the mechanism of AD-MSCs in OA has been explored from the perspective of clinical application [13, 30, 31].

RETRACTED

In our study, we tried to verify the regulatory role of AD-MSCs in the OA model of guinea pigs. During the research, we observed that AD-MSCs were effective in mitigating the gonarthritis of OA guinea pigs, and the overall effect was better than that of SH, a kind of well-accepted therapy for OA [32]. The observation was consistent with current literature that AD-MSCs are a useful method to treat OA [13], especially knee OA [33].

Currently, it is well-recognized that inflammation plays a central role in OA pathogenesis [34]. Here, we discovered the elevation of proinflammatory factors and the decrease of anti-inflammatory factors in the serum and synovial fluid of OA guinea pigs, while the injection of AD-MSCs or SH countervailed the changes. The findings were consistent with the previous discovery that AD-MSCs elicits anti-inflammatory roles in OA [35]. Besides, OA-related factors, including MMP-1, MMP-13 [36], IGF1 [37], ADAMTS4, and ADAMTS5 [38], were all enhanced in the serum and synovial fluid of OA guinea pigs, and AD-MSCs and SH could offset their elevation. However, TGF-*β* expression was higher in both serum and synovial fluid after 3 weeks and higher in the AD-MSCs group and the SH group than that in the NS group. This is possible because active regenerative tissue of the knee joint was often associated with higher levels. The interaction of various cytokines might induce the decline in overall expression in the serum and synovial fluid after 8 weeks.

To unveil the acting therapeutic mechanism of AD-MSCs in OA, we selected OA-related genes from GEO database. Through further qRT-PCR analysis, we focused on BTG2, a significantly downregulated gene in the articular cartilage from OA guinea pigs. BTG2 has been reported as a tumor suppressor to regulate many biological processes in cancers [39]. Moreover, BTG2 has been identified as an inflammation-related gene [40]. Notably, a former report also suggested that BTG2 is one of the candidate genes related to methotrexate resistance in patients with rheumatoid arthritis [41].

BTG2 has been demonstrated to protect human mammary epithelial cells from oxidative stress [42]. Furthermore, Imran and Lim have revealed that oxidative stress could elevate BTG2 expression and finally regulating various biological cell phenotypes [43]. RNA-induced oxidative stress is closely related with disease progression [16, 17]. In this study, we evaluated the ROS level and SOD concentration in the chondrocytes of the OA model with BTG2 overexpression. We uncovered that BTG2 overexpression reduced the ROS level but enhanced the SOD activity suggesting that BTG2 might suppress oxidative stress in OA.

RETRACTED

The current study is the first one to detect the role of BTG2 in OA. BTG2 plays as a molecular switch for the transformation from cell proliferation to differentiation by controlling the exit of a cell cycle as well as the subsequent terminal differentiation [44]. It has a vital role in the maturation of stem cells [45]. Another research showed that the increased stem cells differentiation percentage into neural lineage cells was accompanied by an increasing BTG2 expression level [46]. In our current study, we revealed that activation of the BTG2 molecular switch caused more stem cells to transform from proliferation to differentiation, ultimately resulting in an improved differentiation percentage into cartilage cells. According to the expression level of BTG2, it also increased in AD-MSCs.

Transcription factors (TFs) are one of the main regulators for the critical genes. KLF4 is an evolutionarily conserved zinc finger-containing transcription factor that modulates diverse cellular processes such as cell growth, proliferation, and differentiation [47]. Moreover, KLF4 has already been proven to work as a suppressor of OA progression [26, 27]. KLF4 enhanced expression of major cartilage extracellular matrix (ECM) genes and SRY-box transcription factor-9 and suppressed mediators of inflammation and ECM-degrading enzymes [48]. Another study viewed that KLF4 was negatively modulated by miR-7 and KLF4 was downregulated in human OA tissues and OA chondrocyte [27]. Similar research found that lncRNA MEG3 can promote chondrocyte proliferation and inhibit inflammation by sponging miR-9-5p to induce KLF4 expression [49]. Here, we predicted KLF4 as a potential upstream regulator for BTG2 in OA. We demonstrated the transcriptional activation of KLF4 on BTG2. Our findings about the relationship between KLF4 and BTG2 in OA suggested a potential novel regulatory pathway in OA progression.

In conclusion, our study revealed that AD-MSCs exert effective therapeutic effects on the gonarthritis depending on the upregulation of KLF4-regulated BTG2. Based on plenty of research work, bone marrow or adipose tissue-isolated MSCs have shown great potential for cartilage repair in clinical trials. The findings of current study can help provide some theoretical guidance for the treatment of AD-MSCs on OA.

However, limitations in the current study remain ineligible. First, the mechanism of AD-MSCS-mediated transcriptional activity of KLF4 remains to be investigated. Second, the intercellular molecular transmission which affected the OA progression need to be further explored. Importantly, lack of investigation on clinical samples is also a major limitation of our current study. Therefore, we will further explore these mechanisms in our future study and validate relevant molecular mechanism in clinical samples.

RETRACTED

## Figures and Tables

**Figure 1:** AD-MSCs are effective in treating guinea pig model of OA. (a) AD-MSCs marked with CFDA were observed through *in vivo* bioluminescence imaging. (b) Four different groups of OA guinea pigs treated at the 3^rd^ and the 8^th^ week were subjected to bipedal balance pain testing, with the pain scores of animals in four groups calculated. The sample number for control group at three weeks and eight weeks is separately 24 and 12; the sample number for other three groups at three weeks and eight weeks is separately 54 and 24. (c) The articular cartilages of guinea pigs from indicated groups were photographed, and the damages were scored. *N* = 4 in control group; *N* = 8 in other three groups. ^∗^*P* < 0.05.

**Figure 2:** The MRI results of knee joints from OA guinea pigs. (a and b) At the 3^rd^ and the 8^th^ week after indicated injections, MRI was applied to observe the knee-joint of guinea pigs from indicated groups. *N* = 4 in the control group; *N* = 8 in other three groups.

**Figure 3:** AD-MSCs have therapeutic effects on the gonarthritis of OA guinea pigs. (a) HE staining was utilized to measure the articular cartilage tissues from guinea pigs in four groups (NS, SH, AD-MSC, and control) at the 3^rd^ week and the 8^th^ week after indicated treatments. *N* = 4 in the control group; *N* = 8 in other three groups. All left images: scale bar = 100 *μ*m. All right images: scale bar = 20 *μ*m. (b–d) Safranin O-fast green staining (All left images: scale bar = 100 *μ*m. All right images: scale bar = 20 *μ*m), toluidine blue staining (All left images: scale bar = 100 *μ*m. All right images: scale bar = 20 *μ*m), and sirius red staining (scale bar = 25 *μ*m) of the articular cartilage tissues from guinea pigs in the four groups at the 3rd and 8th weeks after indicated treatments. *N* = 4 in the control group; *N* = 8 in the other three groups. (e) Immunocytochemistry was conducted to examine the expression of Col2 in indicated articular cartilage tissues. *N* = 4 in the control group; *N* = 8 in other three groups. All left images: scale bar = 100 *μ*m. All right images: scale bar = 20 *μ*m.

**Figure 4:** The effects of AD-MSCs on the changes of inflammatory-associated cytokines. (a–l) ELISA examined the content of inflammation- and OA-related factors, including IL-1*β*, TNF-*α*, IL-1, IFN-*γ*, IL-13, TGF-*β*, IL-4, IGF1, ADAMTS4, ADAMTS5, MMP-1, and MMP-13 in the synovial fluid of articular cavity obtained from guinea pigs in four groups (NS, SH, AD-MSC, and control) after 3 or 8 weeks of injections. Number of replicates. *N* = 4 in the control group; *N* = 8 in other three groups. ^∗^*P* < 0.05.

RETRACTED

**Figure 5:** BTG2 is significantly downregulated in the articular cartilage of OA guinea pig. (a) GEO database was applied to predict OA-related genes through common selection of GES12021, GSE55235, and GES55457 with logFC < (-1.0) and *P* < 0.05. (b) qRT-PCR was used to examine the expression of the nine selected genes (GRB10, BTG2, APOLD1,KLF9, MCL1, VEGFA, SIK1, GADD45B, and TNFAIP3) in the OA group (*n* = 8) compared with the Sham group (*n* = 4). (c) BTG2 expression in the articular cartilage obtained from guinea pigs in four groups (NS, SH, MSC, and control) after 3 or 8 weeks of injections. *N* = 4 in the control group; *N* = 8 in other three groups. ^∗^*P* < 0.05. ^∗∗^*P* < 0.01. (d) Western blot assay was conducted to verify the protein level of BTG2 among the different animal groups in different time point. *N* = 3 in each group.

**Figure 6:** KLF4 activates BTG2 expression in AD-MSCs. (a) Potential TFs for BTG2 were selected out through intersecting hTFtarget prediction subset with GEO datasets GES12021, GSE55235, and GES55457 (*P* < 0.05, logFC <0). (b) BTG2 expression was examined by qRT-PCR in chondrocyte separately transfected with overexpression vector of four indicated TFs. *N* = 3 in each group. (c) qRT-PCR examined the expression of BTG2 after KLF4 silencing. *N* = 3 in each group. (d) ChIP assay was conducted to examine the binding of KLF4 to BTG2 promoter. IgG served as a negative control. *N* = 3 in each group. (e) The binding sites of KLF4 in the BTG2 promoter were predicted through the JASPAR tool. (f) Luciferase reporter assay was conducted to prove the binding fragment that was responsible for the interaction between KLF4 and BTG2 promoter. *N* = 3 in each group. (g) DNA pulldown assay was conducted to verify the affinity of KLF4 to BTG2 promoter. *N* = 3 in each group. ^∗^*P* < 0.05. ^∗∗^*P* < 0.01. (h) Western blot assay was conducted to verify the protein level of KLF4 among the different animal groups in different time point. *N* = 3 in each group.

**Table 1:** Macroscopic evaluation of cartilage repair.

Criteria	Appearance	Points
Degree of defect repair	In level with surrounding cartilage	4
	75% repair of defect depth	3
	50% repair of defect depth	2
	25% repair of defect depth	1
	0% repair of defect depth	0

Integration to border zone	Complete integration with surrounding cartilage	4
	Demarcating border<1 mm	3
	3/4 of graft integration, 1/4 with a notable border>1 mm	2
	1/2 of graft integration with surrounding cartilage, 1/2 with	1
	a notable border>1 mm	
	From no contact to 1/4 of graft integration with surrounding	0
	Cartilage	

Macroscopic appearance	Intact smooth surface	4
	Fibrillated surface	3
	Small, scattered fissures or cracks	2
	Several, small or few but large fissures	1
	Total degeneration of grafted area	0

Overall repair assessment	Grade I: normal	12
	Grade II: nearly normal	11-8
	Grade III: abnormal	7-4
	Grade IV: severely abnormal	3-0

RETRACTED

## Data Availability

All data was within the manuscript.

## Supplementary Materials

Supplementary 1 Figure S1: (A) The surface antigens of AD-MSCs (Neg CKTL, CD90, CD105, and CD73) were measured by flow cytometry. *N* = 3 in each group. (B) Differentiation to osteoblasts was demonstrated with phase contrast and by Alizarin Red staining, Oil Red staining, and Alcian blue staining. *N* = 3 in each group.

Supplementary 2 Figure S2: AD-MSCs attenuate inflammation in OA guinea pigs. (A-L) ELISA examined the content of inflammation- and OA-related factors, including IL-1*β*, TNF-*α*, IL-1, IFN-*γ*, IL-13, TGF-*β*, IL-4, IGF1, ADAMTS4, ADAMTS5, MMP-1, and MMP-13 in the serum of articular cavity obtained from guinea pigs in four groups (NS, SH, AD-MSC, and control) after 3 or 8 weeks of injections. *N* = 4 in the control group; *N* = 8 in other three groups. ^∗^*P* < 0.05.

Supplementary 3 Figure S3: BTG2 suppresses oxidative stress. (A) ROS production was detected in chondrocytes of the OA model transfected with pcDNA3.1 empty vector or BTG2 expression vector by flow cytometry. (B) SOD production was measured in chondrocytes with BTG2 overexpression. *N* = 3 in each group. ^∗∗^*P* < 0.01.

Supplementary 4 Figure S4: graphical abstract. A graphical abstract was plotted to illustrate the functions and mechanism of AD-MSCs in OA.
